# Antidepressant-Like Activity of YL-0919: A Novel Combined Selective Serotonin Reuptake Inhibitor and 5-HT_1A_ Receptor Agonist

**DOI:** 10.1371/journal.pone.0083271

**Published:** 2013-12-18

**Authors:** Hong-xia Chen, Zeng-liang Jin, Li-ming Zhang, Rui Xue, Xiao-dan Xu, Nan Zhao, Zhi-kun Qiu, Xian-wang Wang, You-zhi Zhang, Ri-fang Yang, Yun-feng Li

**Affiliations:** 1 Department of New Drug Evaluation, Beijing Institute of Pharmacology and Toxicology, Beijing, P. R. of China; 2 Department of Pharmacology, School of Basic Medical Scieneces, Capital Medical University, Beijing, P. R. of China; 3 Department of Anesthesiology, Chinese PLA 309 Hospital, Beijing, P. R. of China; 4 Department of Medicinal Chemistry, Beijing Institute of Pharmacology and Toxicology, Beijing, P. R. of China; Peking University, China

## Abstract

It has been suggested that drugs combining activities of selective serotonin reuptake inhibitor and 5-HT_1A_ receptor agonist may form a novel strategy for higher therapeutic efficacy of antidepressant. The present study aimed to examine the pharmacology of YL-0919, a novel synthetic compound with combined high affinity and selectivity for serotonin transporter and 5-HT_1A_ receptors. We performed in vitro binding and function assays and in vivo behavioral tests to assess the pharmacological properties and antidepressant-like efficacy of YL-0919. YL-0919 displayed high affinity in vitro to both 5-HT_1A_ receptor and 5-HT transporter prepared from rat cortical tissue. It exerted an inhibitory effect on forskolin-stimulated cAMP formation and potently inhibited 5-HT uptake in both rat cortical synaptosomes and recombinant cells. After acute p.o. administration, very low doses of YL-0919 reduced the immobility time in tail suspension test and forced swimming test in mice and rats, with no significant effect on locomotor activity in open field test. Furthermore, WAY-100635 (a selective 5-HT_1A_ receptor antagonist, 0.3 mg/kg) significantly blocked the effect of YL-0919 in tail suspension test and forced swimming test. In addition, chronic YL-0919 treatment significantly reversed the depressive-like behaviors in chronically stressed rats. These findings suggest that YL-0919, a novel structure compound, exerts dual effect on the serotonergic system, as both 5-HT_1A_ receptor agonist and 5-HT uptake blocker, showing remarkable antidepressant effects in animal models. Therefore, YL-0919 may be used as a new option for the treatment of major depressive disorder.

## Introduction

Major depression is the one of the most common psychiatric diseases with a life-time prevalence of 15–20%, and is predicted to increase from fourth to second (first in high income countries) highest global burden of disease by 2030 [1], [2]. Selective monoamine uptake inhibitors are being used as principle therapeutic agents in the treatment of depression [3]. Among those, especially serotonin transporter (SERT) and norepinephrine transporter (NET) blockers have been used in the therapy for depression [4], [5]. Tricyclic antidepressants developed earlier acted by enhancing both serotonin and norepinephrine transmissions [6]. However, due to their nonspecific interactions with multiple central nervous system (CNS) receptors, they exhibit unwanted side effects which limit their use in the clinics [7]. Development of selective serotonin reuptake inhibitors (SSRIs) alleviated many of the side effects exhibited by traditional tricyclic antidepressants and thus proved to be more effective [8], [9]. However, full efficacy is only apparent after several weeks, and many patients only partially respond, and some remain refractory. Accordingly, considerable efforts are invested in the search for better drugs for more effective treatment of depression.

Several compounds that target 5-HT_1A_ receptors including pindolol and buspirone, have been used to accelerate or enhance the antidepressant effect of SSRIs. Pindolol preferentially competes with endogenous 5-HT at presynaptic 5-HT_1A_ receptors to increase serotonergic neurotransmission [10], [11], [12]. Pindolol has reported to accelerate the antidepressant effect of SSRIs, even in drug-resistant depression [13], [14]. Buspirone functions as strong 5-HT_1A_ partial agonist that can specifically desensitize 5-HT_1A_ autoreceptor to relieve serotonergic autoinhibition [15]. A number of studies have demonstrated an adjunctive efficacy of buspirone when added to variety of SSRIs, particularly in refractory patient populations [16], [17], [18]. Therefore, an alternative approach is to develop drugs with dual 5-HT reuptake blockade and 5-HT_1A_ receptor agonist actions, which has been termed as serotonin partial agonist-reuptake inhibitor (SPARI), the rationale behind this pharmacodynamic combination is presumably to specific desensitization the somatodendritic 5-HT_1A_ autorecepors and also directly simulate postsynaptic 5-HT_1A_ heteroreceptors, and therefore presumably increase serotonergic neurotransmission. A number of molecules combined 5-HT_1A_ agonist and SSRI have been developed, and Vilazodone is the first compound that was approved on 21 January 2011 by the US Food and Drug Administration (FDA) for the treatment of Major Depressive Disorder (MDD). The efficacy data for Vilazodone appears comparable to other known antidepressants, but potentially with a lower incidence of sexual side effects and weight gain. Vilazodone may hold promise for patients who cannot tolerate or have not responded to previous antidepressant monotherapies. Additionally, its use may extend to the treatment of other mental health conditions similar to those treated by serotonin selective reuptake inhibitors [19], [20], [21].

Based on the above mentioned factors, we designed and synthesized a series of compounds with novel structures and activities of both 5-HT_1A_ receptor agonist and SSRI, and YL-0919 [(1-(1-benzyl-4-hydroxypiperidin-4-ylmethyl)-2(1H)-pyridinone hydrochloride, Figure 1A] was screened as the final candidate because of its previously demonstrated antidepressant effects [22]. The frontal cortex is implicated in a number of higher cognitive functions as well as processing emotions and regulations of stress responses, and 5-HT_1A_ receptors are found in high concentration in this encephalic region [23]. In the present study, the binding and function of YL-0919 were measured using 5-HT_1A_ receptor/serotonin transporter binding, monoamine uptake, and cAMP assays *in vitro*. The animal models commonly used to evaluate potential antidepressants, i.e., tail suspension (TST) in mice, forced swimming test (FST) in mice and rats, and chronic unpredictable stress (CUS)model of rats, were used to evaluate the antidepressant effect of YL-0919. Taking into account the relationship between the molecular targets and the therapeutic effect, the present study aims to investigate the involvement of 5-HT_1A_ receptor in the antidepressant-like effect of YL-0919 *in vivo*. Our results may provide a theoretical basis and new avenue for future development and clinical implication of antidepressant compounds.

**Figure 1:** The intrinsic functional activities of YL-0919 on 5-HT_1A_ receptor. **A.** The chemical structure of YL-0919. **B. C. D.** cAMP assays. Both 8-OH-DPAT (10^−11^∼10^−6^ M) and YL-0919 (10^−11^∼10^−6^ M) concentration-dependently inhibited forskolin-stimulated cAMP formation (B). WAY-100635(0.1 µM) markedly prevented the 8-OH-DPAT (10^−11^∼10^−9^ M) (C) and YL-0919 (10^−11^∼10^−9^ M) (D) mediated inhibition of forskolin-stimulated cAMP formation. PC12 cells expressing 5-HT_1A_ receptors were incubated in the presence of 0.5 mM IBMX, 10 µM forskolin and, different concentrations of drugs. Data (presented as mean ±SEM) were representative of four distinct experiments performed in triplicate. **p<0.01 versus the same concentration of 8-OH-DPAT or YL-0919.

## Materials and Methods

### Ethics Statement

All animal experiments were carried out in accordance with the National Institute of Health Guide for the Care and Use of Laboratory Animals (NIH publication No. 86-23, revised 1996). This study was proved by Beijing Institute of Pharmacology and Toxicology. All efforts were made to minimize the number of animals used and their suffering.

### Animals and housing

Male Sprague Dawley rats weighing 180–220 g and male ICR mice weighing 18–22 g (Beijing Vital River Laboratory Animal Technology Company, Beijing, China) were used for the experimental procedure. The animals were group-housed in polypropylene cages under standard experimental conditions: room temperature 22±2°C, humidity 40–60%, 12 h:12 h light/dark cycle (lights on at 8:00 a.m.). Food and water were available *ad libitum*. Animals were allowed to have an acclimation period before each experiment.

### Materials

YL-0919 was synthesized in our institute (white powder with purity >99.8%). Fluoxetine, desiparmine, 8-OH-DPAT, WAY-100635, citalopram, reboxetine, and nomifensine were purchased from Sigma-Aldrich (St. Louis, MO, USA). [^3^H]-WAY-100635, [^3^H]citalopram, [^3^H]8-OH-DPAT, [^3^H]nisoxetine, [^3^H]win35428, and [^3^H]5-HT were purchased from PerkinElmer Life Sciences (NEN, Boston, MA, USA). Dulbecco's modified Eagle's medium (DMEM) and fetal bovine serum (FBS) were purchased from Invitrogen Inc. (Grand Island, NY, USA) and HyClone Corp. (South Logan, UT, USA) respectively. Unless specified below, all compounds were dissolved in distilled water and administered s.c. or p.o. in a volume of 10 mL/kg (mice) or 2 mL/kg (rats)

### Evaluation of the efficacy of YL-0919 on 5-HT_1A_ receptors

#### Evaluation of YL-0919's affinities to 5-HT_1A_ receptors and other binding sites

Male SD rats were killed by cervical dislocation, and the frontal cortex was dissected and homogenized in 40 volumes of ice-cold buffer (50 mM Tris–HCl buffer pH 7.4). The homogenates were centrifuged at 40,000 g for 10 min at 4°C. The pellet was gently resuspended and centrifuged again. Membranes prepared in this manner could be stored at −80°C for up to 1 week.

To assess the binding affinity of YL-0919 to 5-HT_1A_ receptor from rat frontal cortex, competitive binding assays were performed as previously described [24], using [^3^H]WAY-100635 (1.2 nM) as radioligand, and 8-OH-DPAT (10 µM) as non-specific ligand. The radioactivity was determined by liquid scintillation counting. The specified parameters are listed in Table 1. The binding assays were performed in duplicate in three independent experiments. Standard protocols were used to determine the affinities to other potential binding targets, including D_1_, D3, D2, D4, D5, 5-HT_1B_, 5-HT_1D_, 5-HT_2A_, 5-HT_2C_, 5-HT_3_, 5-HT_5A_, 5-HT_6_, 5-HT_7_, α_1A_, α_1B_, α_2A_, β_1_, M_1_, M_2_, M_3_, M_4_, M_5_, μ, κ, δ, A_1_, A_2A_, H_1_, H_2_, H_3_, and H_4_.

**Table 1:** The specific parameters in binding and uptake assays.

Assays	Species	Tissue	Radioligand(nM)	Non-specific ligand(μM)	Reaction conditions
5-HT_1A_ receptor binding	Rats	Frontal cortex	[^3^H]WAY-100635 (1.2)	8-OH-DPAT(10)	37°C,30 min
SERTs binding	Rats	Frontal cortex	[^3^H]citalopram (1.2)	Fluoxetine(10)	37°C,30 min
NETs binding	Rats	Frontal cortex	[^3^H]nisoxetine (1.0)	Desipramine(10)	25°C,60 min
DATs binding	Rats	Striatum	[^3^H]win35428 (1.0)	Nomifensine(10)	25°C,60 min
5-HT uptake	Rats	Frontal cortex	[^3^H]5-HT(20)	Citalopram(10)	37°C,10 min
	cell line	HEK293 cell line transfected hSERT	[^3^H]5-HT(50)	Fluoxetine(10)	37°C,10 min
cAMP assay	cell line	PC12 cell line transfected 5-HT_1A_ receptor	−	−	37°C,15 min

#### Determination of the intrinsic activity of YL-0919 by cAMP assay in PC12 cells transfected with mouse 5-HT_1A_ receptor

PC12 cells stably expressing the mouse 5-HT_1A_ receptor were precious gifts from Dr. Zhi-qing Xu (Capital Medical University, Beijing, China) [25]. These cells were cultured in DMEM supplemented with 2 mM glutamine, 1 mM pyruvate, and 10% heat-inactivated FBS. Subcultures were made by digestion with 0.025% trypsin in PBS, and the cultures were maintained at 37°C in an air/CO_2_ (95∶5) water saturated atmosphere.

The LANCE cAMP kit (PerkinElmer, Zaventem, Belgium) was used to determine cAMP concentrations according to the manufacturer's instruction [26], [27]. Briefly, the cells were grown to 80% confluence, harvested with versene, and washed once with HBSS. The cell suspension was then added to 384-well microplates and preincubated with YL-0919 at concentrations ranging from 10^−11^ to 10^−5^ M for 15 min at 37°C. All experiments were performed in the presence of 0.05% bovine serum albumin (BSA), 0.5 mM of the phosphodiesterase inhibitor isobutylmethylxanthine (IBMX), and 10 µM of adenylcyclase activator forskolin. A “no cell” control and a cAMP standard curve were prepared in parallel. The plates were read at 665/615 nm by EnVision multilabel plate reader (PerkinElmer, Zaventem, Belgium). The results calculated from 665/615 nm ratio were expressed as the percentage of the inhibition of forskolin-induced cAMP production. The specified parameters are listed in Table 1. The cAMP assays were performed in duplicate in three independent experiments.

### Transporter binding and uptake assays

#### The binding of YL-0919 to rat SERTs, NETs, and DATs

The frontal cortex and striatum membranes were prepared as mentioned above. The binding affinities of YL-0919 to rat SERTs, NETs, and DATs were determined by competition with [^3^H]citalopram (1.2 nM, for SERT), [^3^H]nisoxetine (1.0 nM, for NET), and [^3^H]win35428 (1.0 nM, for DAT). Non-specific binding was determined using fluoxetine (10 µM), desipramine (10 µM), and nomifensine (10 µM) for SERT, NET, and DAT, respectively. The binding assays were performed in duplicate in three independent experiments [40]. All specified parameters are listed in Table 1.

#### Upatake of [^3^H]5-HT in rat cortex synaptosomes and human recombinant cells

[^3^H]5-HT uptake assays in rat cortex synaptosomes were performed as described previously [28]. Briefly, the animals were killed, and the frontal cortex was dissected and homogenized in 15 volumes of ice-cold sucrose (0.32 M). The homogenates were centrifuged at 2,000 g for 10 min at 4°C; the supernatants were centrifuged again at 4,800 g for 15 min, and the final pellet was resuspended with 4 mL ice-cold assay buffer (10 mM HEPES, 133 mM NaCl, 4.85 mM KCl, 1.2 mM KH2PO4, 1.5 mM MgSO4, 1.5 mM CaCl_2_, and 11.1 mM Glucose; pH 7.4). The crude synaptosomes were incubated in Krebs buffer containing drug solution and [^3^H]5-HT (20 nM; PerkinElmer, Zaventem, Belgium) at 37°C for 10 min. Non-specific uptake for SERT was determined using 10 µM citalopram. All specified parameters are listed in Table 1. The uptake assays were performed in duplicate in three independent experiments.

The uptake of 5-HT into HEK293 cells stably expressing hSERT was determined using the methods described previously [29]. Briefly, the medium was removed from cells, which were then washed with phosphate-buffered saline. Total 100 µL of Krebs–Ringers–HEPES buffer containing various concentrations of drugs were added into the 96-well plate, and [^3^H]5-HT (50 nM) was added and incubated for 10 min at 37°C. Non-specific uptake was determined using 10 µM fluoxetine. The uptake assays were performed in duplicate in three independent experiments. The specified parameters are listed in Table 1.

### Behavioral studies

#### TST in mice

To determine the antidepressant-like activity of YL-0919, mice were subjected to the TST. The duration of immobility induced by tail suspension was measured according to the method described previously [30] with minor modification. Briefly, 60 min after p.o. drug administration, the mice were suspended on the top of apparatus by adhesive tape placed approximately 1 cm from the tip of the tail. The duration of immobility in the last 4 min of total 6 min suspension was recorded. The immobility was defined as absence of any limb or body movements, except for those caused by respiration.

#### FST in mice

The test was conducted according to the reported methodology originally described by Porsolt et al. with minor modification [31]. Briefly, 60 min after p.o. drug administration, the mice were individually forced to swim in an open cylindrical container (diameter 10 cm, height 25 cm, containing 19 cm of water maintained at 25°C). The duration of immobility in the last 4 min of total 6 min test was recorded. Mice were considered immobile when they ceased struggling and remained floating motionless in the water, making only those movements necessary to keep their head above water.

To investigate the possible involvement of 5-HT_1A_ receptors in the effect of YL-0919 in TST and FST, mice were treated with WAY-100635 (0.3 mg/kg, s.c.) in combination with YL-0919 (1.25, 2.5 mg/kg, p.o), and the TST or FST was carried out 60 min later. The dose of WAY-100635 used was based on the literature [32].

#### FST in rats

The test was performed as described previously [33]. The procedure consisted of pretest and test two sessions, with the same apparatus and condition (diameter 18 cm, height 40 cm, containing 23 cm of water maintained at 28°C). The rats were exposed to a pretest swim session for 15 min 24 h prior to the 5-min swim test session. The duration of immobility in the 5 min was recorded. The criterion for immobility was the same as that described for mice. The drugs were administered p.o. 23 h and 1 h before the test session.

#### Locomotor activity assay with open-field test (OFT)

In order to rule out any non-specific locomotor effect of YL-0919 on antidepressant-like activity, mice and rats were administered with the same regimen as in TST and FST. The locomotor activity was assessed in an OFT. Mice and rats were placed in the corner of the plastic box (the floor was divided into nine equal sectors; 36×29×23 cm for mice, 76×76×46 cm for rats) for 5-min acclimation, then the number of squares crossed with all paws (crossings) and raising the forepaws (rearings) were recorded in the next 5 min session. The square arena was cleaned with a solution of 10% alcohol and dried after each test in order to hide animal cues to prevent from the odor influence by the previous animals [40].

#### CUS model

To further evaluate the antidepressant-like effect of YL-0919, CUS model was applied in rats as described previously [34], [35]. After 1-week acclimation, the animals were subjected to one period of 48-hr sucrose training and several periods of sucrose baseline test. The rats were divided into five groups randomly based on their sucrose preference in the final sucrose baseline test: control (non-stress), stress-vehicle (distilled water), stress-fluoxetine (10 mg/kg), and stress-YL-0919 (1.25 or 2.5 mg/kg). The vehicle or drugs were administered orally during 8:00 to 9:00 am, 1 h before the stress procedure. Except for control non-stressed group, other animals were subjected to stressors as the following: 1) food or water deprivation (24 h); 2) low-intensity stroboscopic illumination (100 flashes/min); 3) overnight illumination; 4) soiled cage (200 mL water in 100 g sawdust bedding); 5) forced swimming (5 min at 10°C); 6) white noise (approx. 110 dB); 7) 45°C cage tilt; 8) tail pinch (1 min); and 9) restraint (2 h). The stressors were applied continuously and randomly as described in Table 2. The rats in control group were left undisturbed in the home cages, except for the 14-hr period of water deprivation prior to each sucrose test. After 4-week stress, OFT, sucrose preference test, and novelty-suppressed feeding (NSF) test were performed without acute drug treatments. The outline of design for CUS and behavioral test is shown in Figure 2A.

**Figure 2:** The effects of YL-0919 in rats exposed to 4-week stress procedure. **A.** The outline of design for CUS and behavioral tests. **B.C.** The effects of YL-0919 and fluoxetine on the number of crossing and rearing. The number of crossing and rearing in stress-vehicle group were significantly decreased after 4-week exposure to chronic unpredictable stress. Daily oral administration of YL-0919 (1.25 or 5 mg/kg) and fluoxetine (10 mg/kg) reversed the inhibition of locomotor activity in CUS rats. **D.E.** The effects of YL-0919 and fluoxetine on the sucrose preference in rats before (D) and after (E) 4-week stress procedure. Four-week stress procedure caused significant decrease in sucrose preference in stress-vehicle rats compared to control non-stressed rats. Four-week treatment of YL-0919 (1.25, 2.5 mg/kg, p.o.) and fluoxetine (2.5 mg/kg, p.o.) restored the sucrose preference to normal level. **F.** The effects of YL-0919 and fluoxetine on the latency to begin eating in rats exposed to 4-week stress regime. Long-term treatment of YL-0919 (1.25 or 2.5 mg/kg, p.o.) and fluoxetine (10 mg/kg, p.o.) significantly reduced the latency to begin eating compared with vehicle-stressed rats. Flu, fiuoxetine. Fluoxetine or YL-0919 was administered p.o. prior to stress procedure. Data are presented as means±SEM (n = 8–11/group). **p<0.01, ***p<0.001versus control, ^#^ *p*<0.05, ^##^ *p*<0.01, ^###^ *p*<0.001 versus stress.

**Table 2:** The chronic unpredictable stress regime.

	Week			
	Week1	Week2	Week3	Week4
Sunday	Tail pinch: 1 min	Overnight illumination: 12 h	Force swimming: 5 min	Overnight stroboscopic: 12 h
Monday	Water deprivation: 24 h	Cage tilt: 24 h	Food derivation: 24 h	Soiled cage: 24 h
Tuesday	Overnight stroboscopic: 12 h	Restraint: 2 h	Overnight illumination: 12 h	Force swimming: 5 min
Wednesday	Soiled cage: 24 h	Tail pinch: 1 min	Restraint: 2 h	White noise: 1 h
Thursday	Force swimming: 5 min	Overnight stroboscopic: 12 h	Water deprivation: 24 h	Overnight illumination: 12 h
Friday	White noise: 1 h	Water deprivation: 24 h	Overnight stroboscopic: 12 h	Food derivation: 24 h
Saturday	Food derivation: 24 h	White noise: 1 h	Tail pinch: 1 min	Cage tilt: 24 h

The locomotor activity of animals was assessed by OFT after 4 weeks of stress procedure. The apparatus was an area 122 cm in diameter with a white, opaque wall 45 cm high, which was divided into 16 sectors. Rats were placed in the center of the arena 24 h after the last drug treatments, and the numbers of crossing and rearing were recorded simultaneously within 5 min.

#### Sucrose preference test

Sucrose preference test [36] was employed in this study to measure the anhedonia, one of the core symptoms of major depression in human. The rats were trained to consume 1% (w/v) sucrose solution for 48 h without food and water supply. Three days later, after 14 h food and water deprivation, 1 h baseline test was performed, in which rats could select between two preweighed bottles, one with 1% sucrose solution and the other with tap water. The sucrose preference (SP) was then calculated as SP = sucrose intake×100%/(sucrose intake+water intake). Following exposure to 4-week stress, sucrose preference test was employed again to evaluate the CUS model and drug action.

#### NSF test

The NSF test was performed according to Bodnoff et al. [37] with minor modification. Briefly, rats that had been fasted for 48 h were placed in the corner of the plastic box (76×76×46 cm) with 12 food pellets weighed approximately placed in the center. The latency to begin eating within 5 min was recorded (defined as the rat chewing or biting the pellet, instead of merely sniffing or toying with it). Moreover, home-cage food consumption in 5 min was immediately evaluated to assess the effect of drugs on feeding drive.

### Statistical analysis

All data were expressed as mean±SEM. The statistical analysis was performed using GraphPad Prism v5.02 (GraphPad Software, La Jolla, CA, USA). The receptor binding and monoamine uptake data were analyzed using one-site nonlinear regression of concentration–effect curve. The Ki values were calculated using Cheng–Prusoff equation: Ki = IC_50_/[(L/Kd)+1], where the IC_50_, L, and Kd are the half maximal inhibitory concentration, the substrate concentration, and the dissociation constant of radioligand, respectively. Two-way analysis of variance (ANOVA) followed by Bonferroni's test was performed in the cAMP assays. As for data from behavioral assays, Student's *t*-test was carried out to compare the difference between two groups; other data were analyzed using one-way analysis of variance (ANOVA) followed by Dunnett's test.

## Results

### Radioligand binding Studies

Radioligand binding assays were conducted to determine the affinity of YL-0919 to rat 5-HT_1A_ receptors, SERTs, NETs, and DATs. The affinity constants (Ki) of YL-0919 were compared with 8-OH-DPAT and those for known antidepressants under identical conditions in the same laboratory. 8-OH-DPAT (Ki = 0.06±0.01 nM), a 5-HT_1A_ receptor full agonist, was one order of magnitude greater than that of YL-0919 (Ki = 0.19±0.02 nM). YL-0919 (Ki = 0.72±0.10 nM) was at the same order of magnitude as fluoxetine (Ki = 0.48±0.01 nM) for SERTs. The affinity constants of comparators were similar to previous studies [38], [39]. The results showed that YL-0919 bound to 5-HT_1A_ receptor and serotonin transporter with high affinity, but its affinity to NET and DAT were low, blocking [^3^H]nisoxetine and [^3^H]win35428 binding with K_i_ values of 650±12 nM and 2652±112 nM respectively (Table 3). To determine whether YL-0919 might also bind to other potential targets, we tested its binding capacity to numerous protein targets including G-protein coupled receptors, such as D_1_, D3, D2, D4, D5, 5-HT_1B_, 5-HT_1D_, 5-HT_2A_, 5-HT_2C_, 5-HT_3_, 5-HT_5A_, 5-HT_6_, 5-HT_7_, α_1A_, α_1B_, α_2A_, β_1_, M_1_, M_2_, M_3_, M_4_, M_5_, μ, κ, δ, A_1_, A_2A_, H_1_, H_2_, H_3_, and H_4_ (data not shown). Except for 5-HT_1A_ receptor and SERT, YL-0919 did not show affinity to any other tested targets, suggesting that the bindings of YL-0919 to SERT and 5-HT_1A_ receptor are selective.

**Table 3:** The affinity of YL-0919 to 5-HT_1A_ receptor and monoamine transporters.

			K_i_ values (nM)	
	Radioligand	Tissues	YL-0919	Comparator
5-HT_1A_ receptor	[^3^H]8-OH-DPAT	Frontal cortex	0.19±0.02	0.06±0.01 (8-OH-DPAT)
SERT	[^3^H]citalopram	Frontal cortex	0.72±0.10	0.48±0.01 (Fluoxetine)
NET	[^3^H]nisoxetine	Frontal cortex	650±12	0..54±0.03 (Reboxetine)
DAT	[^3^H]win35428	Striatum	2652±112	0.23±0.01 (Nomifensine)

The respective K_i_ values(nM) for inhibiting the binding of [^3^H]-8-OH-DPAT, [^3^H]-citalopram, [^3^H]-nisoxetine, and [^3^H]-win35428 to 5-HT_1A_ receptor and monoamine transporters by YL-0919 and other reference agents indicate that YL-0919 bound to 5-HT_1A_ receptor and serotonin transporter with high affinity. The K_i_ values (presented as mean±SEM) were calculated from three independent experiments on different days, and each concentration was run in triplicate.

### [^3^H] 5-HT uptake studies

Consistent with its potent affinity to rat SERTs, the IC_50_ values of YL-0919 inhibiting the uptake of [^3^H]5-HT into rat cerebral cortical synaptosomes and human recombinant cells were 1.78±0.34 nM and 1.93±0.18 nM respectively, while the corresponding IC_50_ values for the reference compound fluoxetine inhibiting the uptake of [^3^H]-5-HT into rat cerebral cortical synaptosomes and human recombinant cells were 32.62±2.74 nM and 49.39±2.04 nM respectively, 18- and 25-fold higher than those of YL-0919 respectively (Table 4). The potency of reference compound fluoxetine, an SSRI, to block the uptake of 5-HT in this study is consistent with previous studies [39], [40].

**Table 4:** The functional properties of YL-0919 and fluoxetine on SERT.

Measurement	IC_50_ values (nM)	
	YL-0919	Fluoxetine
[^3^H]-5-HT uptake-synaptosome	1.78±0.34	32.62±2.74
[^3^H]-5-HT uptake-human recombinant cells	1.93±0.18	49.39±2.04

Both YL-0919 and fluoxetine inhibited the uptake of [^3^H]-5-HT into rat cerebral cortical synaptosomes and HEK293 cells stably expressing hSERT. The IC_50_ values were presented as mean±SEM of three independent experiments performed in triplicate.

### cAMP assays

The 5-HT_1A_ receptor couples to Gi/Go proteins and inhibits adenylyl cyclase activation, reducing cAMP levels in most cells. The intrinsic functional activities of YL-0919 on 5-HT_1A_ receptor were assessed in PC12 cells stably expressing mouse 5-HT_1A_ receptor *in vitro*. While the 5-HT_1A_ receptor agonist 8-OH-DPAT exerted a concentration-dependent inhibitory effect on cAMP formation with an IC50 of approximately 16.4 nM, a similar inhibition was also observed with YL-0919 with an IC50 of approximately 23.9 nM (Figure 1B). In antagonism studies, WAY-100635 (0.1 µM), which failed to show any intrinsic effect by its own, markedly prevented the 8-OH-DPAT- and YL-0919-mediated inhibition of forskolin-stimulated cAMP formation (Figure 1C, *p*<0.01; Figure 1D, *p*<0.01).

### Antidepressant-like effect of YL-0919 in TST and FST

The clinically effective antidepressant drugs SSRI fluoxetine (30 mg/kg, p.o.) and tricyclic antidepressant desipramine (30 mg/kg, p.o.) as positive control caused a significant reduction in the immobility time in TST and FST as compared with vehicle (Figure 3A, *p*<0.001; Figure 3B, *p*<0.01; Figure 3C, *p*<0.001), indicating that the behavioral tests performed under normal condition were reliable. YL-0919 (1.25, 2.5, and 5 mg/kg, p.o.) significantly reduced the immobility time in TST in mcie (Figure 3A, *p*<0.01), FST in mice (Figure 3B, *p*<0.01) and FST in rats (Figure 3C, *p*<0.001), with U-shaped dose-response curves.YL-0919 (0.625-5.0 mg/kg, p.o.) displayed no effect on the locomotor activity of both mice and rats in a separate OFT (Table 5). Furthermore, as shown in Figure 4, the antidepressant-like effect of YL-0919 in TST (Figure 4A, *p*<0.01) and FST (Figure 4B, *p*<0.01) in mice was completely bunted by coadministration with WAY-100635 (0.3 mg/kg, s.c.) that alone did not induce any significant changes in immobility time compared with control group (Figure 4A, *p*>0.05; Figure 4B, *p*>0.05), demonstrating the dependence of YL-0919 function on 5-HT_1A_ receptor.

**Figure 3:** The effect of YL-0919 in the behavioral despair paradigms. YL-0919 produced antidepressant-like effects in TST in mcie (A), FST in mice (B) and FST in rats (C). Veh, vehicle; Flu, fluoxetine; DIM, desipramine. YL-0919, fluoxetine, or desipramine was administered p.o. 60 min prior to the test. Data are presented as means±SEM (n = 10–12/group). *p<0.05, **p<0.01, ***p<0.001 versus vehicle.

**Figure 4:** The effect of 5-HT_1A_ receptor in the antidepressant-like of YL-0919. Coadministration with WAY-100635 (0.3 mg/kg, s.c.) prevented YL-0919 (1.25, 2.5 mg/kg, p.o.)-induced reductions in the immobility time in TST (A) and FST (B) in mice. WAY, WAY-100635; YL, YL-0919. Mice received WAY-100635 and YL-0919 simultaneously; 60 min later, the animal were submitted to the forced swimming. Data are presented as means±SEM (n = 10/group). **p<0.01, ***p<0.001 versus vehicle, ^##^ *p*<0.01 versus the same dose of YL-0919.

**Table 5:** The effect of YL-0919 on locomotor activity in mice and rats.

Species	Dose of YL-0919(mg/kg)	Locomotor activity	
		No. of crossing	No. of rearing
Mice	0	84.4±6.7	19.7±1.8
	0.625	87.8±6.4	19.3±2.2
	1.25	82.1±5.0	22.2±1.7
	2.5	81.3±6.6	20.0±1.9
	5.0	83.3±5.5	19.8±1.5
Rats	0	62.6±6.0	15.3±1.4
	0.625	66.3±5.1	14.6±2.1
	1.25	61.7±4.8	15.4±1.6
	2.5	59.4±5.3	16.1±2.1
	5.0	60.9±4.7	14.8±1.7

YL-0919 displayed no effect on the locomotor activity of both mice and rats in OFT for 5 min. YL-0919 was p.o. administered 60 min before OFT. Data are presented as means±SEM (n = 10/group).

### The effect of YL-0919 on CUS rats in OFT

The locomotor activity of CUS rats was observed in OFT. The numbers of crossing and rearing in stress-vehicle group were significantly reduced after 4-week exposure to CUS (Figure 2B, *p*<0.01; Figure 2C, *p*<0.001), while daily oral administration of YL-0919 (1.25 or 2.5 mg/kg) reversed the inhibition of locomotor activity in CUS rats, evidenced by markedly increased numbers of crossing and rearing compared with stress-vehicle CUS rats(Figure 2B, *p*<0.01; Figure 2C, *p*<0.01), consistent with the effect of the reference antidepressant fluoxetine (10 mg/kg), which also significantly increased the number of crossing and rearing in CUS rats(Figure 2B, *p*<0.05; Figure 2C, *p*<0.05).

### The effect of YL-0919 on sucrose preference in CUS rats

As shown in Figure 2D, following sucrose training and baseline test, the intakes of sucrose and water were basically stable, and the sucrose preference in all groups was similar before stress regime. The 4-week stress procedure resulted in a significant decrease in sucrose preference in stress-vehicle rats compared to control non-stressed rats (Figure 2E, *p*<0.001), while the treatment with YL-0919 (1.25 or 2.5 mg/kg) clearly restored the sucrose preference to normal level (Figure 2E, *p*<0.001). The reference antidepressant fluoxetine treatment (10 mg/kg, p.o.) also significantly increased the sucrose preference level in CUS rats (Figure 2E, *p*<0.001).

### The effect of YL-0919 on latency to begin eating in CUS rats

The NSF test has been demonstrated to be sensitive to chronic antidepressant treatment [41]. Figure 2F shows the effect of YL-0919 on CUS rats in NSF test. Compared to control non-stressed rats, 4-week stress procedure significantly increased the latency to eat in stress-vehicle rats (*p*<0.01), while long-term treatment with YL-0919 (1.25 or 2.5 mg/kg, p.o.) significantly reduced the latency to begin eating compared with vehicle-stressed rats(*p*<0.01)., which is in consistence with the effect of positive control, fluoxetine (10 mg/kg, p.o.), which significantly reduced the latency to begin eating in CUS rats too (*p*<0.05). However, there was no difference in the home-cage food consumption among groups (data not shown).

## Discussion

In the present study, we performed pharmacodynamic and pharmacological evaluation of YL-0919, a structurally new compound with high affinity at both 5-HT_1A_ receptor and 5-HT transporter, and demonstrated that YL-0919 exerted a significant antidepressant-like effect after acute and chronic administration in various mouse and rat models.

The receptor binding studies demonstrated that YL-0919 displayed high affinity for rat 5-HT_1A_ receptor and serotonin transporter, whereas showed low affinity to NET, DAT, and other G protein coupled receptors, suggesting the dual-target binding profile of YL-0919. The functional characterization of YL-0919 binding to 5-HT_1A_ receptors was carried out *in vitro* with a cell line stably expressing the receptor by analyzing its ability to inhibit forskolin-stimulated cAMP formation. The concentration-dependent inhibition of cAMP formation by full agonist 8-OH-DPAT was blunted by simultaneous application of WAY-100635, results in keeping with previous studies [42]. Similarly, a low concentration of YL-0919 also exerted a concentration-dependent inhibitory effect on cAMP formation, which can be markedly blocked by coadministration with WAY-100635 too. These results indicate that in this assay, YL-0919 eventually behaves as a 5-HT_1A_ receptor agonist.

The results obtained from neurotransmitter uptake assays showed that in accordance with its affinity to SERT, YL-0919 potently inhibited the uptake of [^3^H]5-HT into rat cortical synaptosomes, and this effect was 18-fold more potent than that of fluoxetine. Similar results were also obtained with recombinant cells, where YL-0919 exhibited a 25-fold greater efficacy than fluoxetine. The potency of fluoxetine, as positive control, to block the uptake of 5-HT in this study is consistent with previous studies [39], [40]. These functional assays indicate that YL-0919 acts as a 5-HT uptake inhibitor.

Behavioral despair paradigms played an important role in the evaluation and development of antidepressant drugs. The TST in mice and FST in mice and rats are among the behavioral models that are widely and routinely used to screen new antidepressant compounds for their ease of use, reliability, specificity, high predictability of clinical efficacy [43], and generally high sensitivity to 5-HT_1A_ receptor agonists [44]. The present study has shown that very low doses of YL-0919 significantly reduced the immobility time in these behavioral despair models with U-shaped dose-response curves. These results from TST and FST in mice and rats were similar to those shown with conventional SSRIs, i.e., fluoxetine in TST (30 mg/kg, p.o.), and tricyclic antidepressants, i.e., desipramine in FST (30 mg/kg, p.o.), but at a much lower dose (1.25, 2.5, and 5 mg/kg, respectively, p.o.); such doses were similar to those of Vilazodone [21]. The results obtained from all three behavioral despair paradigms in mice and rats clearly demonstrated the antidepressant-like efficacy of YL-0919. In the TST and FST, false-positive results may exit with certain drugs, in particular, psychomotor stimulants, which also could decrease immobility time by stimulating locomotor activity [45]. To rule out non-specific motor effects of YL-0919, locomotor activity of mice and rats was evaluated at the same dose that showed antidepressant-like effect in the TST and FST. YL-0919 did not increase locomotor activity, indicating that the antidepressant effect of YL-0919 was not associated with stimulating motor activity.

Although multiple 5-HT receptors may be involved in antidepressant behavioral responses, the activation of 5-HT_1A_ receptors appears to be important for SSRIs to exert behavioral effects in antidepressant test [46]. It has been reported that treatment with 5-HT_1A_ receptor antagonists or genetic deletion of 5-HT_1A_ receptor could totally prevent the behavioral effects of SSRIs [41], [47]. In accordance with the agonist activity of YL-0919 on 5-HT_1A_ receptors, the antidepressant-like effect of YL-0919 was completely blocked by WAY-100635, suggesting that YL-0919 exerts its antidepressant-like effects mainly through the activation of 5-HT_1A_ receptor. However, whether YL-0919 acts on presynaptic autoreceptors or postsynaptic 5-HT_1A_ receptors need further studies. It should be noted that only further studies using, e.g., electrophysiological [48] or voltammetric method, can finally confirm this interpretation [49], which our group is currently working on.

The CUS model has been widely used in pre-clinical antidepressant evaluation. It is well reported that stress is one of the major risk factors provoking depressive disorder. CUS model induces a variety of behavioral deficits and neurochemical or neuroendocrine disturbance, which is in accordance with clinical symptoms or alterations in depressive patients [34], [50]. In this study, 4-week stress induced a significant reduction in both locomotor activity and sucrose preference, which were indicators of the core symptoms of major depression, i.e., lack of reactivity and anhedonia. Concomitant YL-0919 administration restored these behavioral deficits to a normal level, suggesting its antidepressant-like activity and in agreement with its acute action. Furthermore, it has been documented that the CUS model may also induce anxiety-like symptoms [51], [52]. The NSF test was initially used to examine the effects of anti-anxiety agents [34]. Acute and chronic treatment with anxiolytics or chronic treatment with antidepressants significantly reduces the first latency for animals to eat in novel environment. In this study, 4-week stress resulted in a prolonged latency to eat, which was reversed by chronic YL-0919 treatment. Take all the behavioral results into account, we conclude that YL-0919 applied either acutely or chronically, displays a definite antidepressant-like activity in multiple animal models in mice and rats.

The greater increase of 5-HT levels in vitro induced by YL-0919 in comparison with fluoxetine is similar to the augmentation effects achieved by Vilazodone campared with fluoxetine in the ventral hippocampus and the frontal cortex using in vivo microcdialysis [53]. However, Vilazodon does not display any advantage over existing post-tricyclic antidepressant [54]. In the present study, YL-0919 and fluoxetine behave similar in the behavioral despair paradigms and rat stress model. Another compound, VN2222, with a dual action at 5-HT_1A_ receptors and 5-HT transporter also showed similar antidepressant-like effect in the learned helplessness tests in rats [55], [56]. The dose of YL-0919 exerting antidepressant-like effect was similar to that of Vilazodone and VN2222 [21], [55], [57], but YL-0919 in this study represents another novel class of antidepressant compounds with a totally different chemical molecular structure. Moreover, compared to the vilazodone with complicated structure and hard to dissolving in water, it can be easily synthesized and dissolved in water; metabolic studies have also shown that its concentration reaches the micromolar level in mouse and rat brain tissues after taking the prototype of YL-0919.

In summary, this work has presented a novel compound, YL-0919, acting as both serotonin specific reuptake inhibitor and 5-HT_1A_ receptor agonist. Such pharmacological profile of dual functions may account for its antidepressant-like activity demonstrated in animal models. Future studies are needed to further assess the feasibility of its clinical application in eliciting an efficacious antidepressant response in patients.
